# Blockchain-Based Land Registration System: A Conceptual Framework

This article has been retracted.

**DOI:** 10.1155/2022/3859629

**Published:** 2022-02-15

**Authors:** Muhammad Irfan Khalid, Jawaid Iqbal, Ahmad Alturki, Saddam Hussain, Amerah Alabrah, Syed Sajid Ullah

**Affiliations:** ^1^Department of Information Technology, University of Sialkot, Pakistan; ^2^Department of Computer Science, Capital University of Science and Technology, Islamabad, Pakistan; ^3^Department of Information Systems, College of Computer and Information Sciences, King Saud University, Riyadh 11543, Saudi Arabia; ^4^School of Digital Science, Universiti Brunei Darussalam, Jalan Tungku Link, Gadong BE1410, Brunei Darussalam; ^5^Department of Information and Communication Technology, University of Agder (UiA), N-4898 Grimstad, Norway

## Abstract

Land registration authorities are frequently held accountable for the alleged mismanagement and manipulation of land records in various countries. Pakistan's property records are especially vulnerable to falsification and corruption because of the country's poverty. Different parties therefore claim varying degrees of authority over a specific piece of land. Given the fact that this data has been consolidated, it has become significantly more vulnerable to security threats. The goal of decentralized system research has been to increase the reliability of these systems. In order to fix the flaws of centralized systems, blockchain-based decentralized systems are currently in development. By using significant land record registration models as the basis for this research, we hope to create a proof-of-concept system or framework for future use. Pakistan's land registration agency will benefit from our proposed conceptual framework. For the Pakistani government to implement a decentralized land record registry system, we propose a conceptual framework that outlines the essential components.

## 1. Introduction

The process of land registration in any country is known to be a multistep process, since it entails the engagement of all stakeholders who will have a direct or indirect stake in the registration. The currently used land record title storage system raises major issues about data fraud, the security of highly sensitive data, and the risk of system failure due to natural disasters, such as the server used for data storage going down [1]. Compared to the current approaches and procedures for land title management and data storage, blockchain is a cutting-edge technology and database that has the ability to completely address the problems that plague current systems. The basic and most important aspect of blockchain technology is that it is a decentralized network in which all data supplied by a single node are confirmed by all other available nodes, and only after a consensus is made can then the shared data be saved to the blockchain [2].

There are various platforms being used for the creation of reliable, decentralized, transparent, immutable, and secure blockchain-based land registration and management systems. Smart contracts based on the Ethereum blockchain are gaining traction among these systems. Being a public blockchain platform, it allows anyone to participate in the blockchain ecosystem [3].

Many attempts have been made to map the land records to this emerging technology (blockchain) with the goal of securing and maintaining land data. In this regard, the UAE was one of the countries that took the initiative and developed a strategy for incorporating blockchain into their projects. The Dubai Land Record Authority was one of the first government agencies to put its land titles on the blockchain [4]. However, in developing countries like Pakistan, the access to land record as well as the management of data has been a serious concern. In Pakistan, out of four major provinces, i.e., Sindh, KPK, Baluchistan, and Punjab, only Punjab Province land record data has been stored to the computer in Pakistan. In some provinces, land data is still stored and managed typically by a central person known as a “patwari,” who saves this crucial data on big paper-based registries. In this regard, the Punjab government took important measures and built an information system known as the “Punjab Land Record Management Information System,” to simplify the complex process of saving and managing land records [5]. Despite the fact that digitalization of documents and other related data has speed up the process, security, resilience, and traceability remain important concerns. Due to a lack of infrastructure for the land registry system, property records are particularly vulnerable to inconsistent, inaccurate, and tampered data.

Blockchain technology offers decentralized environment that is reliable and secure. The process of the land management and title recording system is being used for storing land title facts and running the transactions that are intertwined in land titles. Since these records are sensitive, land management and title cataloging systems must be robust in order to prevent falsification, make these records available at all times, and, most importantly, complete these operations in a timely manner [6]. Blockchain is no longer limited to simple principles; it has evolved into a hybrid of several replicas, including mathematics, networking, cryptography, and a distributed consensus algorithm [7].

Blockchain was developed from bitcoin paper published by Nakamoto in 2008. It is a peer-to-peer network where all participants (peers) serve as a node and all the nodes hold the same information [8]. Blockchain is a ledger dispersed publicly above a network that registers transactions associated bordered by other network applicants [9]. Instead of relying on the single authority such as administrators that can forge the database, blockchain technology offers decentralized environment that offers robustness and security as well. Untrustworthy administrators can abuse this power. A normal database suffers from that issue which is the failure that occurs at a single point, and it makes them to depend much on backups if some failure occurs. Moreover, due to this failure if both, i.e., backups and an operating database are abused, it is catastrophic [10].

The process of the land management and title recording system is being used for storing land title facts and running the transactions that are intertwined in land titles. As these records are sensitive, land management and title cataloging processes should be strong in order to avoid falsification, making these records available all the time, and more importantly, these processes should be completed in a very short span of time [11]. The functionality of blockchain also considered a digital register. Blockchain-based land registry schemes use the same functionalities as sound land registry systems have. At the same time, blockchain knows that these assets are owned by that person and also at what time a particular transaction took place [12].

### 1.1. Motivation and Contributions

Based on the limitations of the central server-based data storage systems for land record data of Pakistan, we emanated up with blockchain-based solution that will be able to handle those problems from which the existing centralized land record data storage system is suffering. Digitizing real-world land records require systems to be built which are robust and can withstand hacking attempts. Such systems need to be built upon frameworks that can ensure integrity and longevity. No such frameworks exist for implementing a blockchain-based land registry system in Pakistan, which can be used for a real-world implementation of a decentralized land record registry. The systematic contribution is to offer a significant and authenticated conceptual framework for blockchain-based land registration systems where transparency, security, and rights can be made sure without the need of the trusted third party. A centralized server for land record data is facing numerous issues, i.e., loss of data due to any natural hazards and loss of data due to some strong adversary that can forge all the available data. Among all these concerns, the most bulging and pragmatic problem is that the land record officials who are dealing with the data can also counterfeit the data and many stakeholders who are the actual owners of a piece of land can be unable to find their authentic rights. In this contribution, our major concerns are to make the official of the government be aware about the potential of one of the most disruptive technologies, i.e., “blockchain,” and at the same time to reflect the issues that current land manipulation systems are facing. Our motivation and goal are to give a solution to the centralized land management system shortcomings using distributed and decentralized blockchain technology. For this, first we proposed a blockchain-based conceptual framework and then validated that framework with the blockchain-based proof-of-concept system (PoC). We first used Ethereum blockchain to validate our framework and then discussed and did few experiments on the idea of moving land record data to the blockchain technology with the government officials and those who are currently using centralized Punjab land record authority systems.

In this paper, we have contributed towards the research community as follows:

- We observed the evident flaws in the current land registry systems of Pakistan and presented a study that gave meaningful insights into the adoption of blockchain technology
- We discussed and disseminated the required information with the concerned stakeholders, i.e., land registration authority officers who are the ultimate users of the current centralized system and future blockchain-based land registry system
- We have done experiments for showing the effectiveness of our study along with the potential of one of the disruptive technologies, i.e., “blockchain”
- Our study will prove to be the first drop of rain in bringing transparency and security to the sensitive land record data and its manipulation procedures

### 1.2. Related Works

A record keeping system is based upon blockchain, and it removes the vulnerabilities to the sensitive data. It is because of this reason that blockchain uses cryptographic primitives for the process of authentication. That is why blockchain can be used to reduce the trust on the third party by decreasing cost through the process of a programmed transaction recording system [13]. Those applications that are being controlled and managed by the single or central user are called centralized applications. In centralized applications, all the parties reconcile their local databases with a centralized electronic ledger that is maintained and controlled by a trusted central party. Moreover, record keeping has always been a centralized process that always requires trust in the record keepers. Blockchain technology, which has been widely used for the design of decentralized currencies, self-extracting digital contracts and intelligent assets over the Internet, can serve as a replacement for centralized control over records [14].

Centralized systems are numerous, and today's world is the world of social networking. Social networking platforms like Google and Facebook have created the revolutionary connection in humanitarian society. Also, with these platforms, it also made it great responsibility to manage user privacy and one's data that are very much vital for him. In these social networking systems, there lies a central server where all their data reside [15]. Please see Figure 1 for depiction.

In a centralized system, there is a central or single control that manages all the events and coordinates with the whole system. In contrast, in a decentralized system, every participant/entity is completely self-directed. In this autonomous system, each entity is referred to as a peer. In a more comprehensive way, we can say that instead of a centralized system, the use of a decentralized system is becoming mandatory, because everyone wants security, traceability, and resilience in their system. And these emerging technologies like blockchain can play their part to accomplish this much needed task [16]. As the time has passed and new trends have been settled in the technology stack, blockchain has also got more and more attention. Now, it is being used in almost every organization of the government and supply chain and in many other numerous areas. Blockchain has smoothed the problematic, time-consuming processes that were at the risk of failure. In simple words, it has made human more powerful towards the implementation of transparency and accountability and in maintaining trust and security. In this decentralized system, there is no intermediary intervention and the system can be evaluated for the required performance [17]. Please see Figure 2 for the elaboration of decentralized systems.

Every technology will have its own limitations and problems/issues. Though decentralized systems have given strong support to manage security, still these systems are facing problems. For instance, there is an increase in blockchain (emerging decentralized technology) usage and the volume rise in the number of transactions occurs on a daily basis. Due to the variations in the size of each block, in the same way, the time to produce a novel block becomes a primary cause of the not reacting behavior of blockchain [18]. Another rising issue of decentralized systems is the leakage of transaction privacy; this happens because details of the public keys are visible to each participant that is available on the blockchain network [19]. Apart from the advantages of the technologies, there exist few or more cons too; on the one side, blockchain is improving the current state of almost every aspect of data storage and security. It also suffers from few prevailing and alarming problems. In the same way, decentralized systems, i.e., blockchain, are also facing the fork problem. The problem of forks mainly occurs when blockchain is divided into two branches; it can happen due to the change in the consensus algorithm or when there happen some changes to the software. These two problems are directly related to the blockchain's architecture. Normally when there is a change in the consensus algorithm, the soft fork takes place, as at this point the older nodes of the blockchain are unaware about the consensus rule changes. This soft fork can be harmful to the effectiveness and stability of the network. On the other hand, hard fork condition occurs, in decentralized systems when there is a permanent divergence in the blockchain, and this happens when the old nodes have not upgraded themselves to the newer version, and as a result, they cannot validate the transactions [20].

### 1.3. Existing Land Record Management System of Pakistan

In Pakistan, land record data are still being stored either on a centralized server or on paper-based huge registers that are being monitored by a single person who is known as patwari. Although the government has taken steps in digitization of land record, still many land data need to be saved onto a computer which is a centralized server in nature. This centralized server can become a single point of failure, i.e., due to attacks of hackers and due to environmental factors, and the person who is managing and overseeing the complete system can also forge the data [21]. Now, when we talk about land or land titles, there comes a question in everyone's mind as these are the heaps of records that are very abundantly sensitive and vibrant at the same time. And how one can achieve this whole record? The answer to this question is to have land registries that are intended to manage and organize to store land record data in a normal and appropriate way. In a land registration process, one can save the data of those who are going to sale or purchase the pieces of land. This can also be termed as an official and standard record system where anyone can get his/her land information. Land registration, at a wide range, describes systems for defining the ownership rights over the permanent property while the information concerning the property and land-related rights is usually protected and regulated by the government [22].

The process of storing land record data onto a computer is called digitization. The process of digitizing land records was accepted with the intent to reduce flaws in the record keeping systems. In this, process all the records, i.e., sales, purchase, information about the land, and information about the current and former ownership stored in a centralized system. The system was expected to greatly lessen the number of land disputes, as fake documents would be hard to come by and would have little legal use [23]. The elaboration of the fard issuance process can be seen in Figure 3.

In Pakistan, in provisional bodies, i.e., Punjab, the land record data is managed by the Punjab Land Record Authority (PLRA). We have added the complete process of land record registration in Pakistan, and below are steps with the figures. The complete procedure of land registration consists of four steps, and they are as follows:

- Fard issuance
- Fee pay process
- Hiring of a deed writer/lawyer
- Registrar office process

### 1.4. Fard Issuance

Fard is the process that is used in the verification of an individual who has applied for the land transfer, ownership, and purchase. It is a thirty-minute process. It mainly involves the following steps:

- Authentication from NADRA (National Database Regulatory Authority)
- Checking the land and those who have the rights of a piece of land
- Issuance of fee challan
- Submitting fee for their land registration
- And finally issuance of a fard for further proceedings

### 1.5. Fee Paying Process

After getting the fard document from the first phase, the next step is to pay fee in order to process your registration to the next phase. Usually, it takes one day to verify the fee submission process. It mainly involves the following steps: please see Figure 4 for details about the fee paying procedures.

- Get challan from the PLRA website
- Pay fee in the any branch of Bank of Punjab
- Pay challan
- Receipt of stamp paper

### 1.6. Hire a Deed Writer or Lawyer

In this step, the customer now will hire any lawyer or deed writer in order to write the details of the customer that will be submitted to the registrar office for the final verification.

### 1.7. Registrar Office Process

After getting the services of a deed writer, customer application for the land registration will be forwarded to the registrar office. Here, the customer will submit all the documents. The registrar office is the central body in the whole land registration process. This process will check all the steps that have been passed previously, and that is the reason why this is an eight-day process. This process consists of the following steps: Figure 5 is explaining this process.

- Required document submission to the registrar office
- Stamp paper verification and fee processing
- Fard online verification
- Electronic capturing of deed details
- Approval of registry of the subregistrar
- Scanning of past registry and online transmission to the Arazi Record Center
- Automatic attestations of mutation by assistant director land record

### 1.8. Process of Data Entry into the PLRA System

Finally, the service of entering data into the system is the main constituent in the development of a mechanized land record system. The complete process of data entry in the centralized system is described here; in this process, there are multiple steps that are dependent on each other. While there is an internal validation included that led to the removal of errors that occur during the record saving to the system, the whole systems seem to be dependent upon the human intervention and scanning and copying the documents. Please see Figure 6 for data entry procedures into PLRA.

1. Rights that can be registered

The rights in rem that can be registered are ownership, rights of use and residence, land transfer, afflictions, leases, debts, right of recovery, and other rights.

(2) Requirement of the title that can be registered in the land register

For the title to be registered, they must be recorded in a public deed or an authentic document issued by the government under the rules and the prescribed regulations of the government. The title would be entered in the deed if it fulfils the requirements of the deed.

(3) List of documents for registration

There are some documents for the land registration:

- CNIC (owner)
- e-stamp paper
- Challan receipt
- Proof of ownership

The registrar does the registration of the title [24].

### 1.9. Blockchain-Based Land Registration

As blockchain offers, security, accountability, and record can be scrutinized from the start to end. In the typical land registration process, there are three main terms used. These are as follows:

- Object (spatial unit or land)
- Right (personnel rights in terms of land)
- Subject (the titleholder of the right that is related to the object)

Across much of the world, the land registries are going to be called “badly kept, mismanaged, or corrupt.” And then, they have started looking towards this technology, i.e., blockchain, and started saying that this technology should have to bring trust and transparency in the systems. There should be traceability and immutability to the records that are going to be mapped with the blockchain [25]. In every system, the administration and registration play an important role in bringing clarity and validity in these systems. In the same way, the management of land records in a compact way brings transparency, immutability, and trust with blockchain technology. A land registering procedure requires the depth understanding of those terms and procedures that were created in the early times, because the identity of a piece of land can be traced through the addresses and details that have been written in the old registers. That is the reason why none should have sound knowledge of this property recording system [26].

Nowadays, various types of blockchain can be found, and these are well known as private and public. There are some other types though, but we were focusing on these kinds of blockchain. Blockchain has been separated into various types as per its functionality and nature. In a public blockchain, every member of the system has full rights and availability and the actors are welcomed to join the whole system without any kind of problem of security. These members of the system can participate in transactions as per their wish, and the rest of the network remained conversant about the variations that these participants are going to make with the system. The use of a public chain is contingent upon the nature of the system or use case on which one is working. If anyone wants to give access to all the members of the system, then this type is more feasible to him [27].

As far as private blockchain is concerned, it is more limited towards specific members of the systems. There is no frankness for all the members of the network; rather, a system admin will add and then one can access the system of private blockchain. As private companies feel that they are not going to share access with all over the system and they still want to use distributed ledger technology in their organization like banks and financial intuition, they are more settled with the private blockchains. Hence, in these kinds of blockchains, there lies a control over inspecting and changing the transactions and these circumstances are predetermined with respect to the roles allocated. Private blockchains are a perfect cause to get benefit from blockchain technology by making some groups and striking verification who can interact with the system [28]. Please refer to Table 1 for the types of blockchains.

The proof of work concept was initially proposed by Nakamoto as we have defined above; the proof of work is mainly covering the mining that majorly includes the confirmation and proof of some sets of transactions or blocks in any network by presentation of the computational proof of work. It is regarded as a set of consensus protocols of blockchain that were presented by the bitcoin, and now they are being used by a number of other cryptocurrencies too [29]. As bitcoin is operated on Ethereum blockchain, in comparison to bitcoin blockchain, Ethereum offers a blockchain-based development stack where decentralized apps can be built. Ethereum has opened a number of chances through its full stack blockchain-based infrastructure for decentralized applications. Bitcoin blockchain is functioned through the proof-of-work consensus protocol while Ethereum is being operated by proof-of-stake or proof-of-concept protocols [30].

The need for legal contracts for the blockchain is provoked when bitcoin blockchain has presented its power to be functioned with any type of peer-to-peer transactions. This was the arrival of smart contracts. Smart contracts are essentially piece of code that typically runs on the top of the blockchain network. In real-time situations, they are rooted on a blockchain node and digital assets are being supervised by the logic that one has embedded in this smart contract [31].

Having satisfied all the above requirements is of no use, if there is absence of trained community that will interact with the blockchain and its processes. Having satisfied all the above prerequisites to implement a blockchain-based system is not enough. If you do not have such individuals who have basic knowledge of such system, then the process can be impractical. That is the reason why most of the companies invest more on their human resource as they must tackle with the circumstances where the company must maintain their integrity and values. The community who is going to work with these blockchain systems should be trained enough so that they may get the understandings about the pros and cons of the process on which they are working. They should be educated about the land registry systems and the technology in which the use case is going to be implemented, i.e., blockchain in our case. In that way, one can deploy such systems in a systematic way [32].

Frameworks always create easiness for the community who is working to explore a new thing. They also gave the support to the concepts that have been constructed for a specific study [28]. In the same way, conceptual frameworks guide the path that a research uses and offer the foundation for establishing its credibility. In many empirical and exploratory studies, conceptual frameworks are the compulsory prerequisite in a thesis or dissertation that shows the student's map of the research he seeks to comprehend [33]. A researcher can seek many benefits from a conceptual framework. In order to formulate his world view on a phenomenon, these frameworks help a researcher to enhance his view more and more in order to inquire certain aspects of a system [30]. The conceptual framework presents a clear image/picture of systems that needs to be built. We can also say that developing a huge system is a much difficult task. Rather when you build a conceptual framework, then it made things more and more evident to be explored and all the required parts of that system become clearly visible. In other worlds, the conceptual framework made researchers to offer their practiced measure to a problem [34].

Conceptual frameworks consist of the main components on which a system should be developed. They also answer the most arising question that why research should be taken into a certain topic. They also depict what a researcher assumes and how he is going to ground his approach conceptually [35]. The thinking of the entire process can be acquired from these conceptual frameworks. Many a time, these frameworks consist of certain diagrams and figures and these are designed to clearly understand the variable of a research topic, and the relationship between the components of conceptual frameworks is shown with the help of arrows [36].

Nigerian tertiary institutions have used blockchain technology for the digitization of the academic records, as all the academic records are being saved in a manual form or in a centralized storage. In addition, security of digitized academic records depends on the accuracy of processing and storage. The Nigerian institute has used time stamps and a digital signature scheme in this proposed framework. This approach has proven as an alternative in the perspective of authoritative access of the database of academic record [37].  Figure 7 is the proposed architecture of academic record security using blockchain.

The auto insurance accountability models are now going to be disrupted by the advent of autonomous vehicles. In this study, they have proposed a conceptual framework that is based upon the permissioned blockchain. The given framework is designed in a way that it combines all the required entities that a liability model should have. In a simplified form, this also explains the main components that an autonomous system must have. In a conceptual framework, the integral part is the communication of its components, so that a complete and detailed system should be developed in the future. Here, in this liability framework, they have also given importance towards the partitioned communication that is being made to guarantee that the data exchange is only based on a need-to-know basis [38]. Please see Figure 8.

Virtual organizations and blockchain are two emerging technologies in which researchers are keen to explore the possibilities to solve problems and challenges. In this regard, for the healthcare system, blockchain is also used to automate the systems of validating healthcare records. In this in-depth study, a conceptual framework has been proposed. This framework has been proposed with the intent to provide a blockchain-based healthcare system that will guide complete steps on how to verify healthcare service providers and how to validate the records [39].  Figure 9 is expounding about the healthcare-based blockchain model.

Blockchain is also being used in public service delivery in Sri Lanka. Three distinct public service delivery systems were analyzed in order to derive a common framework that can be used to design a blockchain-based solution for the public sector processes. Systems were reformed using blockchain technology, and two prototypes were developed using two different present platforms [40].

## 2. Research Methodology and Framework Design

The focus of this study is to explore the current systems and bring innovation by the exploration of these existing systems. Therefore, we adopted exploratory research. Exploratory research methodology is defined as finding out what is happening, seeking new intuitions, and generating ideas and theories for new research. In the first section, we have explored and analyzed what is happening in the land registration process in Pakistan, and from these examination and exploration processes, we have collected new insights. With these new insights, we are in a position to produce some concepts and hypotheses. In the second part, we have explained our experiments that we have done in preparation of this conceptual framework.

### 2.1. Data Collection

In our research, we have applied a primary data collection technique as its best suits the empirical researches and it is usually carried out through either observation or the primary communication with the stakeholders. Here, we have communicated directly with stakeholders and those who are part of the system (land sale and purchase).

### 2.2. Interviews

We have conducted semistructured interviews of ten respondents who were land officers and village officers from Multan and Islamabad and serving in the Punjab Land Record Authority (PLRA).

### 2.3. Document Review

In parallel to an interview approach, we have gone through from the document reviewing process. We have thoroughly reviewed the documents available at the Punjab Land Record Authority for land registration purpose. This technique has been used in order to maximize the diversity of the data.

### 2.4. Data Analysis

For the concrete understanding of the interviews, we have employed a thematic analysis approach. The technique of thematic analysis is a very flexible method of qualitative data analysis. This method is specifically being used for identifying, examining, and reporting all those patterns or themes that are present in the data. In our case, we have collected data in the forms of interviews and employed the thematic analysis approach to draw some important patterns and themes from this collected data. Although thematic analysis itself uses some of other methods for the exploration and detailed information, still we have used an “anything goes” approach as this approach is abundantly being used for the assessment of qualitative data. This “anything goes” approach does not have any strict guidelines in the given method; also, it can be used for any framework, either theoretical or conceptual framework. Moreover, it can be used for the detailed and complete assessments of qualitative data.

### 2.5. Data Coding

Data collected during this research was in semistructured format that makes it difficult to analyze and process further. Therefore, it needs to be consistent and in one single format to be processed by the techniques. For this, we have used the qualitative analysis software CAQDAS (Computer-Assisted/Aided Qualitative Data Analysis Software). We have employed our data to this software. This has made our representation quite understandable. The RQDA tool itself assisted in examining the written data and helped to create codes that were afterward applied to various parts of the records; a code characterized a theme and construct. One code is usually allocated to many pieces of text, and one piece of text can be assigned more than one code; therefore, some parts of the texts, based on the theme, were labelled with several codes and generalized afterwards to draw some logical patterns. Please see Figure 10 for the opted research methodology for this paper.

### 2.6. Proposed Framework and Its Validation

This section details the design of the proposed framework and its basic functionalities along with deployment of different record keeping techniques. We have carried out an empirical study that has shown the importance and need of a blockchain-based system for the sensitive data of land records. Further, the validation of the proposed framework is carried out in two phases, namely, simple smart contract-based blockchain and experiments carried out to collect the data from stakeholders, which are discussed in this section.

### 2.7. Technology Used and the Design of the Framework

As we have discussed earlier, in our framework, we have given access only to those entities that are authorized to interact with the system. In this regard, we have used private blockchain to enhance security, integrity, and traceability of land record data. We have used multichain blockchain (which is a private blockchain) for the formulation of this framework. The complete design of this framework lags this blockchain's permissioned node, i.e., multichain. We have utilized certain protocols of the multichain in order to design this framework as per the needs and the requirements.

### 2.8. Framework Design

The framework has been designed with some entities that will interact with the system. To keep a check on who can interact with the ledger, it is essential to conceptualize using permissioned blockchains. A blockchain node is there that has imparted the permissioned effect in this design. There are actors, and they have their roles in this framework. We have described all the processes of the framework in detail. In the first step, when a user/patwari/village officer will register a piece of land, then he should have to login into the system. After that, he will initiate a request to register this piece of land.

### 2.9. Concepts of Land Registry Systems

If we start from the advent of the record keeping technique, then it is obvious that there was no guarantee that we can certify reliability and trust. There was a single entity named as village officer/patwari who has all the record. What he must do is to write the details of any piece of land on a paper or on the animal's skin. This is known as the “khasra number” that is the point of identification for ownership. With the passage of time when these record keeping techniques gave birth to disputes and corruption, then a digitization process was introduced. Unfortunately, although this has eliminated the forgery and corruption, still it was a centralized storage for the record keeping. In our framework, there are two main concepts: land registry office and land registry officer. The blockchain process after will validate the transaction made by the officer that any transaction/entry can be made to the land registry. This will eliminate the third party that is a patwari or the other concerned person who can forge the land records.

### 2.10. Proposed Framework

Here is our proposed framework for blockchain-based land registry systems.  Figure 11 shows our proposed framework.

#### 2.10.1. Actors and roles

In our proposed framework, there are some actors and they have their roles as well.

#### 2.10.2. Actors

User is a person who will register the title deed of the land known like patwari.

A blockchain operator or block generator will validate the transactions (government officer/officials).

#### 2.10.3. Roles

In our case, there are two actors, i.e., human actor who interacts with the blockchain technology by creating the transactions. This actor is called the “user.” Secondly, we are working with the permissioned blockchain; that is why there exists a blockchain operator that would be a human and he will verify and validate the transaction on the basics of the consensus from all the participants of the network. Here is the complete conceptual framework for the blockchain-based land registry systems. In this proposed system, we have used permissioned or private blockchain that is multichain blockchain, as we did not want to open this to the public. The only people who can look into the system are the registered members. Whenever a user will want to add a block to the blockchain, he must create a transaction for this purpose. When a transaction will be created, then a consensus process will take place as every node of the private blockchain will have a copy of the transaction. When a ping for the transaction takes place, then every node of the block of chain will check the transaction according to the copy that it has. If majority of the blocks verify this, then the consensus will be completed after the verification and validation and the block will be added to the chain. There would be a smart contract that would have an embedded logic in it. When a government official conforms to the transaction, this transaction will be stored onto the blockchain. Please see Figure 12 which is our ultimate proof-of-concept system.

### 2.11. Data block model

Here is a data model; we have used the input and output in order to make sense the complete process of blockchain-based land registries. Here, the block has transaction and the ID of these transactions while the transaction has the update and delete attributes in it. When any block/transaction is not verified, then it will be deleted, others can be validated, and transactions can be updated as the same. The assets or the registry relates to the transactions that will be made in it. The registry will have the name of the landowner, his address, title number of the land, and area of the land. In the same way, the block header will have the address of the last block and timestamp of the block. Please see Figure 11.

The block contains transactions, while the metadata of the block is kept in the block header.  Figure 13 shows the data block model for our proposed framework:

### 2.12. Platform for Validation of the Proposed Framework

#### 2.12.1. Validation Using Simple Blockchain

In the first step, for the validation of this proposed framework, we have used Ethereum smart contracts that depict the real-time working of the land registry on the technology of blockchain. We have done this validation via a private blockchain network where only those participants who can interact with the chain are authorized to do so.

#### 2.12.2. Environment

Above is the remix solidity interface that is showing the validation procedure of the framework; here, we have used smart contract in which all the logics are embedded. A landowner named “ASAD” has a piece of land with the name of “250 shahzad khan.” He has a social security number that is an essential requirement for the land registration system.  Figure 14 shows the environment for the validation process: please see Figure 13 for the testing of our framework using Ethereum blockchain.

### 2.13. Smart contract compiler processing

In Ethereum solidity integrated development environment, there are two steps in the first step; the written smart contract is compiled with the required version of the compiler. In this compilation process, the compiler checks for the possible bug/errors in that written smart contract, and after that, IDE pops up for the next step.  Figure 15 shows the smart contract compilation process: please see Figure 14 for the smart contract compilation representation.

### 2.14. Transaction addition

After the compilation step, the written smart contract is subjected to the final deployment step. Here, the logic embedded in that smart contract is displayed in the form of transaction creation and addition, respectively. For the proper running of this smart contract, we have used a JavaScript virtual machine.  Figure 16 shows the addition of transaction: please see Figure 15.

### 2.15. State transition in blockchain after transaction

When we have added a transaction into blockchain, then the state of blockchain also gets changed. As soon as we have clicked that button “Deploy the contracts,” it changed the state of blockchain and a completely changed interface appeared in order to deploy the contracts to get them verified by the participants.  Figure 17 shows the state transition in blockchain after transaction: please see Figure 16 for the change of states in blockchain.

### 2.16. Transaction validation and block addition process

After the successful running process, a transaction is recorded, i.e., when a user “Muhammad Irfan Khalid” purchases the piece of land. In addition, he is willing to pay the desired price for that piece of land; then, after the verification from the permissioned blockchain node, this transaction is completed and a new person becomes the owner of that piece of land; as a result after this transaction, a fresh block will be boosted to the blockchain.  Figure 18 shows the transaction validation and addition process: please see Figure 17 where transactions are getting validated.

## 3. Evaluation and Findings

### 3.1. Overview

This section has briefly described the experiments and techniques that we have used to validate our proposed framework and results that we have received by doing these experiments. Firstly, we have used a blockchain technology experiment in order to validate the framework. Secondly, we have done an experiment that led us to evaluate our study. For the sake of the evaluation of this framework, we have collected the primary data and then evaluation has been performed because of this data. As we have explained in previous sections that we have used an empirical research method, we have performed some experiment for the sake of validation of our framework. Our proposed framework is the product of the existing frameworks for blockchain-based systems and the response that we have received from the participants.

### 3.2. Validation through PoC Blockchain

In the first phase of validation, we have developed a simple blockchain based on smart contracts. In this validation, we have shown how private blockchain can be used for the land registration system. However, we have designed an extensive illustration of our proposed framework, but still it can be validated with the help of a simple blockchain. We have opted a different technique that was “Ethereum smart contracts with solidity.” We have run few tests using the Ethereum blockchain platform in real-time environment where the ownership of land can be shifted from one person to another. However, it does not happen in a manual way; rather, we have performed with the help of smart contracts. We have registered a piece of land and defined its price as the same. In the next step, we have used logic that was embedded into smart contracts, where when a person wants to buy a piece of land, he must pay the price that was defined by the smart contracts. When the defined price criteria are met after that, a transaction takes place resulting in change of ownership from one person to another.

### 3.3. Results from Blockchain Proof of Concept

This validation through PoC has given us insights that in the future, we can also build such systems where all the functions of land record registries can be fulfilled. Here, we have automated a land sale purchase process and then directed it to the blockchain through smart contract. In this way, the complex data of land record can also be marked as safe as there would be transaction record. The pattern that is currently followed by the higher authorities like PLRA is centralized data storage. The data is being stored in a centralized server. In our case, there is a decentralized data storage system where every single entity should have access to the system as far as the comparison of these two systems is concerned for evaluation; by using the decentralized system, the land record data can be digitized with the blockchain automated process also; by the blockchain immutable process, the security of land record data cannot be compromised easily. In previous studies, there was a great intention to implement blockchain technology in supply chain management, healthcare, and many other fields in Pakistan. However, very few studies are available that has given attention towards the land record systems. We have constructed a framework and gave an idea that these systems can also be built for management of land record registry systems as well. As far as our results are concerned, as we have used exploratory research methodology, we have explored this use case (land registry systems) with the technology (blockchain) and found that if proper attention would be given, then certainly we can have such land registries where there would be trust, security, availability of data, and traceability at the same time. As per the basic functionalities of blockchain after developing such systems, in the future, the land record data would become more reliable, available, and traceable.

### 3.4. Experiment

Apart from the validation that has been discussed in the previous section using blockchain, we have also done an experiment where we have discussed and elaborated the complete procedure of land registration along with the results. We have discussed our proposed PoC with those who are dealing with land registry systems. In this experiment, we have included some of the village officers (patwaris) and those who are currently managing land records, i.e., the staff of the Punjab Land Record Authority (Ali Pur). We have done this experiment with 20 people from district Muzaffargarh and district Rawalpindi, Pakistan. Here, we have divided our experiments into two demonstrations: in the first phase we have given a demonstration to those who have been using the pen and paper system while starting land record data and in the second phase we have done a demonstration with the staff of PLRA.

In the first phase of our experiment, we have described briefly our proposed framework and system where the land registry is supposed to be based upon the technology of blockchain. As in this demo, the majority of our audiences were illiterate or had primary to elementary level of education. We have elaborated on our PoC from the start to end. They have also asked a number of questions on this, and these questions were the base for our results which we have described in detail in the next section. In view of that procedure which they have been using, i.e., saving land data into registers, we have explained our PoC. As we have described in the above section, we have chosen a particular use case where the ownership of the land can be transferred in a real-time environment. We have noted down their feedback about our PoC and their reservations on this PoC as well.

In the second phase of our experiment, we have given another demonstration to the staff of PLRA. The staff of PLRA was adequately educated as compared to those who have been given demonstration in the first phase. Firstly, we have discussed the details; the systems on which the Punjab Land Record Authority is packing land record data are completely centralized, while in our PoC, we have proposed a decentralized system where there is a distributed network. After sharing enough details, we have given them a demonstration where we have shown one of the use cases of land management that was the transfer of the ownership using the blockchain-based land registry system. There, we have shown them how a deed can be covered in a single transaction (as we have shown in our validation section above). After having enough discussion, we have received their feedback which we have written in the next section. We have received both positive and negative feedback on this.

Someone has believed that this technology is far away from our knowledge. As we only know how to click on a URL and print the details of any person who asks for that. In the same way, some people who have been in touch with the latest technologies using smart devices have also given their feedback where they have asked us to implement this in all over the country so that the existing hurdles in the existing system can be abolished in an automated way. With this experiment, we have gathered a number of factors which are a barrier in implanting the latest technologies in a system which is being practiced from the past.

And finally, based on this experiment inputs/feedback, we have concluded the results.

### 3.5. Postexperiment Survey

After having sessions with participants, we conducted a postexperiment survey to record the participant's response and experience about the proposed framework. The postexperiment survey consisted of four questions regarding the proposed framework's feasibility, acceptance, and performance. A total of 20 participants answered these questions, and their responses are rated on the scale of 1 to 5. Please see Table 2.

Participants rated each question based on their experience with a blockchain-based land registration system in which we provided sufficient information and demonstrated the real-time operation of blockchain in which we changed the ownership of land from one person to another using smart contracts.

We have gathered the feedback of the participants on the basis of following these questions:

- Blockchain-based land registry system is feasible
- Blockchain-based land registry system is acceptable to use
- Blockchain-based land registry system eliminates the issues of the existing system
- Blockchain-based land registry system makes the land record management process easy

### 3.6. Postexperiment Results

An experiment with the land record authority and village officers revealed that our land management system still requires some basic improvements. Many of them, with the exception of those who use computer-based work systems, do not have a fundamental understanding of blockchain technology. We then received their feedback on our proposed PoC as well as its use in a real-time context. They were hesitant to deploy the blockchain-based system since the transition from a standard data entry system to a totally decentralized system appeared daunting. If a department has to use blockchain-based solutions, all of its personnel must be completely familiar with them. This can be defined as the employees' learning process as it relates to evolving technologies. We concluded from their response that some fundamental measures should be made before executing or investing in these blockchain-based systems in order to gain acquaintance with these important and growing technologies so that we can implement them in our enterprises. Despite the fact that we showed a demonstration at the conclusion so that they could have a sense of the technology, they were unable to grasp the significance of this PoC. We suggest a private blockchain-based land record management system with access restricted to individuals who work with data in land record offices and those who grant authorization to interact with it. They can monitor land data in real time if they have access to such systems. As previously said, there are some challenges in putting this system into practice in Pakistan. Using a blockchain-based decentralized system necessitates a significant amount of understanding. After that, one can interact with that kind of system. We then received feedback from those with whom we conducted our experiment, including PLRA staff and certain village officers from various places. Please see Table 3.

The blockchain-based land registry system is feasible.

Please see Table 4 for further details about the experimental results of the second question.

Please see Figure 18 for the information of the experimental results of the first question.

The blockchain-based land registry system is acceptable to use.

Please see Figure 19 for the information of the experimental results of the second question.

The blockchain-based land registry system eliminates the issues of the existing system.

Please see Table 5.

Please see Figure 20 for the information about the experimental results of the third question.

The blockchain-based land registry system makes the land record management process easy.

Please see Table 6.

Please see Figure 21 for the information of the experimental results of the fourth question.

## 4. Results and Discussion

The purpose of the above evaluation was to determine the impact of adopting a blockchain-based land registry system for those who are new to it and are now relying on centralized systems for strong land record data. Our evaluation was based on four fundamental questions designed to learn about the participants' perceptions and experiences with a blockchain-based land register system. These questions centered on the first-time user's experience with a decentralized system for managing land records.

There were three research questions in our research:

1. What are the different land registry systems?
2. What are the different frameworks available for blockchain-based systems?
3. What can be the main components of decentralized land registry systems?

We have formulated the outcomes of the validation of our proposed system in light of these research issues. It goes without saying that if industry adopts such frameworks, they can be used to innovate traditional processes. There is comprehensive innovation and advancement for the people, from paper work to the blockchain-based system.

### 4.1. Trust

Our framework is based upon the technology of blockchain; that is why it guarantees trust. Instead of relying on a central entity, our framework puts decentralized trust in the parties involved. Here, there would be complete information about the ownership and the process of the ownership.

### 4.2. Transparency

Each step of the framework is well defined. Anyone can keep track of the changes that have occurred. There is no risk of forgery or corruption because there is no unauthorized access to the system. As stated in the framework, when a transaction occurs, the entire process shall be carried out in complete transparency. We have also looked at the traditional method of storing land records. Similarly, we looked into the current practice of the Punjab Land Record Authority (PLRA). There are significant differences between these two systems, one of which was the one we have proposed here (blockchain-based system). In the existing land record saving method, the seller and buyer must seek authorization from the local managerial organizations. After that, they will be directed to the district and tehsil offices. The whole practice takes up to 10 to 15 working days, and after this stipulated time, one can get the possession of his land. On the other hand, in our proposed system, there is no such type of time and procedure. In our system, there is no central authority; rather, each block participating in the process verifies the transaction. Furthermore, there is no risk of data loss or corruption in a blockchain-based system because blockchain uses a time-stamped method that allows users to follow any data changes. As a result, we may conclude that our proposed approach is far superior to the current standard practices for information storage.

### 4.3. Limitations

Despite the fact that we proposed a framework, our research has some limitations. According to our research, in order to adopt blockchain-based systems, the community that will engage with the system must be capable of managing new technologies, such as blockchain in our case. We inquired about the automated method for recording land records during the study and received a surprise response. We can claim that “change resistance” will be the most challenging obstacle because most of these folks are not computer literate and will find any system with a steep learning curve problematic.

### 4.4. Results of Experiments with Stakeholders

Experiments were conducted to evaluate our proposed conceptual framework using blockchain PoC. These experiments have provided us with both positive and negative feedback on our suggested framework. Participants' responses to using the proposed frameworks were collected in a post experiment survey.

## 5. Conclusion

The paper presents a link to offer a conceptual framework for blockchain-based land registry systems. Following a review of various frameworks, as well as some of the more vigorous approaches and concepts employed in these frameworks, they were mapped with a scenario that led to the conceptual framework. The mapping of the scenarios aided us in classifying the major components, which has been useful to our proposed framework. A land registry combined with blockchain technology has the potential to truly revolutionize governance. After identifying the necessary components, we developed a framework based on fundamental notions that have been employed in both classical and new record keeping systems. Land record storage, like today, has a centralized origin. As a result, this centralized storage can be hacked, forged, or misappropriated, while in our framework, we used entirely decentralized blockchain-based solutions. We have also highlighted privacy as a fair consideration. Some of the nodes in the framework are required as part of the decentralized system's characteristics. Only those who are permitted to interact, such as a block generator or a government official or officer, can interact in this system.

In terms of methodology, we gathered primary data directly from the stakeholders, including government offices and officers, village officers, and the general public who use this system. We conducted semistructured interviews to assess our framework and obtain feedback from both public and government entities.

## 6. Future Work

Currently, we have used a private blockchain-based conceptual framework; however, in the near future, this procedure can be extended to allow the public to connect directly with the system and obtain information about their assets. Furthermore, we have merely been in operation for the purpose of developing a conceptual framework. However, such frameworks can be used to create a software system in the future. As a framework, it can undoubtedly provide insight into the actual system.

## Figures and Tables

**Figure 1:** Centralized application architecture.

**Figure 2:** Decentralized application architecture.

**Figure 3:** Fard issuance.

**Figure 4:** Fee paying process.

**Figure 5:** Registrar office process.

**Figure 6:** Process of data entry into the PLRA system.

**Figure 7:** A blockchain-based conceptual framework for augmenting security of digitized academic records.

**Figure 8:** A blockchain-based framework for liability attribution for autonomous vehicles.

**Figure 9:** Service provider validation and verification framework for the blockchain-based healthcare system.

**Figure 10:** Components of research methodology.

**Figure 11:** Data block model.

**Figure 12:** Proposed conceptual framework.

**Figure 13:** Validation environment.

**Figure 14:** Compilation process.

**Figure 15:** Transaction addition.

**Figure 16:** State transition in blockchain after transaction.

**Figure 17:** Transaction validation and block addition process.

**Figure 18:** Feasibility report of the blockchain-based land registry system.

**Figure 19:** Acceptability of use.

**Figure 20:** Issues in terms of the existing system.

**Figure 21:** Easiness in terms of blockchain.

**Table 1:** Types of blockchain.

Name	Public blockchain (permission less)	Public blockchain (permission less)	Consortium blockchain (permission less)
Access	No access (restrictions)	Invitation only by the network administrator	Restricted to selected consortium members
Transact	Anyone can make transactions	Only those who have rights	Selected consortium members only
View	Anyone can view	Shared between trusted parties	Restricted to selected consortium members
Type	Large, decentralized, i.e., bitcoin and Ethereum cryptocurrency platforms	Middle ground platforms, accounting and record keeping procedures	Participating companies equally involved in the consensus and decision-making

**Table 2:** The participant's response and experience of using the proposed framework's PoC.

Survey questions	Strongly agree (5)	Agree (4)	Uncertain (3)	Disagree (2)	Strongly disagree (1)
Blockchain-based land registry system is feasible	4	9	2	4	1
Blockchain-based land registry system is acceptable to use	3	5	1	6	5
Blockchain-based land registry system eliminates the issues of the existing system	13	4	0	2	1
Blockchain-based land registry system makes the land record management process easy	15	3	0	2	0

**Table 3:** Experiment result 1.

Total participants	Strongly agree	Agree	Uncertain	Disagree	Strongly disagree
20	4	9	2	4	1

**Table 4:** Experiment result 2.

Total participants	Strongly agree	Agree	Uncertain	Disagree	Strongly disagree
20	3	5	1	6	5

**Table 5:** Experiment result 3.

Total participants	Strongly agree	Agree	Uncertain	Disagree	Strongly disagree
20	13	4	0	2	1

**Table 6:** Experiment result 4.

Total participants	Strongly agree	Agree	Uncertain	Disagree	Strongly disagree
20	15	3	0	2	0

## Data Availability

The data used to support the findings of this study are available from the corresponding author upon request.
